The article "The Current Status of SSRP1 in Cancer: Tribulation and Road Ahead" was retracted in 2023. Reasons: unreliable results or conclusions; concerns about the data; concerns about the peer review; concerns about the citations.

# The Current Status of SSRP1 in Cancer: Tribulation and Road Ahead

**DOI:** 10.1155/2022/3528786

**Published:** 2022-04-13

**Authors:** Shengnan Jia, Baofeng Guo, Lihui Wang, Liping Peng, Ling Zhang

**Affiliations:** ^1^Department of Respiratory Medicine, The First Hospital of Jilin University, 71 Xinmin Street, Changchun, Jilin 130021, China; ^2^Department of Hepatopancreatobiliary Medicine, The Second Hospital of Jilin University, Changchun, China; ^3^Department of Plastic Surgery, China-Japan Union Hospital of Jilin University, Changchun, China; ^4^Key Laboratory of Pathobiology, Ministry of Education and Department of Pathophysiology, College of Basic Medical Sciences, Jilin University, 126 Xinmin Street, Changchun, Jilin 130021, China

## Abstract

**Methods:**

We search PubMed and Web of Sciences with keywords “SSRP1” and “Cancer.” Only English literature was included, and conference papers and abstract were all excluded.

**Results:**

Transcription factors are classified into three groups based on their DNA binding motifs: simple helix-loop-helix (bHLH), classical zinc fingers (ZF-TFs), and homeodomains. The tumor-suppressive miR-497 (microRNA-497) acted as an undesirable regulator of SSRP1 upregulation, which led to tumor growth. The siRNA (small interfering RNA) knockdown of SSRP1 hindered cell proliferation along with incursion and glioma cell migration. Through the AKT (also known as protein kinase B) signaling pathway, SSRP1 silencing affected cancer apoptosis and cell proliferation.

**Conclusion:**

The MAPK (mitogen-activated protein kinase) signaling pathway's phosphorylation was suppressed when SSRP1 was depleted. The effect of curaxins on p53 and NF-B (nuclear factor-*κ*B), and their toxicity to cancer cells, is attributable to the FACT (facilitates chromatin transcription) complex's chromatin trapping.

## 1. Introduction

Cancer has been considered the world's second largest reason for death worldwide [1]. The complexity and heterogeneity of tumors have provocation for comprehensive initiatives in cancer diagnosis and treatment [2, 3]. Tumor cell genomic heterogeneity and an environment of proinflammation are important influences in the development of tumors [4, 5]. TNAs, including genes, siRNAs/miRNAs, and oligonucleotides, were delivered to cancer cells, which enabled cancer to be tackled by restored tumor-suppressor expression and silencing oncogenes [6–10].

The key techniques in cancer treatment using nonviral gene therapies are shown in Figure 1. Angiogenesis-targeting therapy, immunization gene therapy, cancer-related fibroblast targeting, and tumor cells-derived exosome targeting are all forms of tumor microenvironment therapies (in green). Genetic strategies include genome editing, miRNA preferential treatment, transcription factor decoys, oncogene silencing, tumor-suppressor gene deletion, and suicide gene therapy (in purple).

The downregulation of specific genes happens as nucleic acids are introduced into tumor cells, a mechanism known as gene silencing [11, 12]. Typically, gene silencing therapy is carried out by vaccinating siRNA or shRNA into tumor cells to mark a particular corresponding classification to RNA (mRNA) of a specific genetic factor, enabling it to degrade or suppress protein synthesis [13, 14].

Ribosomes are protein synthesis catalysts with diverse arrangements that include protein and RNA elements. They are overexpressed proteins in cancer. Eukaryotic ribosomes are classified into two subunits, the 40S and 60S, which are named for their sedimentation coefficients. The small subunit comprises an 18S ribosomal RNA (rRNA) particle and about 33 proteins. The large subunit contains about 49 proteins [15–17]. mRNA and TRNA are connected to the minor subunit throughout protein synthesis, and a large subunit catalyzes the peptide bond. Ribosome catalytic processes are thought to be regulated primarily by rRNA molecules. Many ribosomal proteins may not seem necessary for the operation of ribosomes, and the likely task is to increase the rRNA's function. The ribosomal protein S6's phosphorylation in response to numerous growth factors has been discovered as a growth regulator, whereas some roles of other ribosomal proteins are not recognized [17, 18]. Ribosomal proteins are overexpressed in breast cancer, liver, and colon [19]. Increased cell proliferation or development does not immediately increase ribosomal protein mRNA [20] immediately. In other words, there is valid proof that ribosomal proteins are likely to lead to cell's malignant transformation [21].

Invasive colorectal cancer was first identified to amplify and overexpress ZKSCAN3 (ZNF306 or ZNF309). The investigators found that ZKSCAN3 knockdown in colorectal cancer cells dislocated self-governing development and orthotopic tumor production, while ZKSCAN3 overexpression had the reverse effect [22].

Specific protein-1 (Sp1) was called proponent-specific binding factor needed for SV40 immediate early (IE) gene transcription [23]. Sp1 was once thought to be the general transcript factor used to transcribe many “housekeeping genes,” also known as maintenance genes [24]. Many of the housekeeping genes that are indispensable in cancer instigation and growth have become even more apparent. Sp1 sustains basal levels and a large range of cellular genes, activating and inhibiting them [25, 26].

## 2. Structure-Specific Recognition Protein-1 (SSRP1)

SSRP1 is based on a chromatin transcription facilitated complex (also known as FACTp80) that replicates, transcribes, and repairs DNA. The cell differentiation stage is associated with SSRP1. In proliferation and undifferentiated cells, SSRP1 is highly articulated [27].  Figure 2 shows the STRING interaction network highlighting SSRP1. Transcriptional control, damage repair of DNA, and cell regulation cycle are functions of structural-specific recognition protein-1 (SSRP1) [28]. SSRP1 is overexpressed in several tumor tissues, but is underexpressed in mature tissues [29]. SSRP1 is expressed at significantly elevated levels in multiple human tumor cells [30, 31]. In many cancer-related cases, elevated SSRP1 expression has been linked to metastasized tumors, making SSRP1 a potential prognostic marker and an anticancer target for tumor inhibition [32, 33]. SSRP1 knockdown in colorectal tumors inhibits relocation, propagation, and invasion and encourages apoptosis [34]. FACT aids as a marker and a target for active breast cancer cells [35]. SSRP1 expression is higher in stem cells and cells that are less differentiated, but it is lower in more differentiated cells [36]. The biological activities of SSRP1 are regulated by the HMG domain [37].

## 3. Possible Mechanisms of SSRP1

MicroRNAs (miRNAs) are 18–25 nt noncoding RNAs that bind to the three untranslated regions (UTRs) of target mRNAs to impede translation [38]. MicroRNAs play several roles in the growth of the disease. Tissue morphogenesis, proliferation, and apoptosis are cellular processes that miRNAs play a role in [39, 40]. MicroRNA-28-5p (miR-28-5p) [41] has been shown to suppress tumor growth in several cancers [42], including natural killer lymphoma, hepatocellular carcinoma, and prostate cancer [43–45]. Cheng Wang et al. discovered that miR-28-5p prevents the migration and proliferation of human renal carcinoma cell lines. miR-28-5p blocks the migration of breast cancer cells, according to Liang Ma et al. The miR-28-5p/CAMTAN2 axis controls colorectal cancer development, and miR-28-5p undesirably controls SSRP1 [46]. If the transcription of the mRNAs is decreased, the stability of the protein complex is significantly reduced and its levels rapidly decrease (Figure 3) [47].

According to immunohistochemistry results, downregulation of SSRP1 in xenograft tumors weakens migration and invasion potential in vivo. Organs such as the kidney, heart, lung, liver, and spleen were not affected by SSRP1 knockdown [48]. Diagnosing some diseases, such as heart failure, is a difficult undertaking, much more, so in underdeveloped and emerging nations, human expertise and technology are few [49, 50]. Curaxins, anti-SSRP1 molecules, cause apoptosis in tumor cells [51]. In vivo, silencing SSRP1 activated the AKT signaling pathway, causing downstream apoptosis and cell cycle proteins to alter their expression. In vivo and in vitro, SSRP1 inhibition substantially decreased colorectal cancer proliferation and metastasis and promoted apoptosis [40, 52].

Data show that miR-497 inhibits CCND1 and several other well-studied oncogenic proteins [53]. In most adult tissues, SSRP1 protein levels are modest, but the pathways behind the upregulation of SSRP1 in cancer are still unknown. SSRP1 was miR-497's first direct goal. The miR-497 expression is undesirably associated with SSRP1 expression. SSRP1 is also implicated in cancer cell chemosensitivity. It indicates that miR-497 downregulation can play a role in cancer cells developing a chemoresistance phenotype [54, 55]. Phosphor-Ets-1 translocation from the cytoplasm to the cell nucleus is assisted by SSRP1. The expression and phosphorylation of Ets-1 were only slightly influenced. Ets-1 is a positive regulator of Pim-3 [45]. Docetaxel treatment after SSRP1, Ets-1, or Pim-3 knockdown on apoptosis, inhibition of incursion, and clonogenicity in HNE-1 cells were not effective as NPC cell proliferation, apoptosis, autophagy, incursion, and clonogenicity have all been linked to SSRP1/Ets-1/Pim-3 signaling in the past. Docetaxel chemosensitivity in cells is increased when this signaling is blocked [56, 57]. A previous study reported that active DNA demethylation by DME needs SSRP1 function through a distinct process from direct DNA methylation control (Figure 4) [58].

## 4. Role of SSRP1 in Various Tumors

In the following, we discussed the role of SSRP1 in some well-developed tumors. We highlight the recent progress with recent challenges in each cancer and future perspectives.

### 4.1. Hepatocellular Carcinoma (HCC) and SSRP1

Protein expression and its levels in HPA, SSRP1, and mRNA were significantly higher in HCC than in normal liver tissue [59]. Furthermore, in HCC patients, higher SSRP1 expression was linked to shorter survival and progression-free survival period. As a possible prognostic marker, SSRP1 needs further clinical research. SSRP1 prevents acute lipid catabolism cycles, inflammatory reactions, and peroxisome structure [34, 60]. The molecular mechanism of HCC carcinogenesis is dependable with these results. SSRP1 affects immune cell infiltration, which facilitates the production of HCC and can influence the impact of immunotherapy [59, 61]. In transgenic mice expressing the Her2/neu protooncogene, FACT expression upregulated during tumorigenesis of mammary carcinoma in vivo. The mRNA and protein levels are upregulated in HCC [62]. The upregulation of SSRP1 may help the accumulation of DNA and gene mutations in HCC cells. In HCC, SSRP1 was discovered to be an oncogene. After curative hepatectomy, it could be a new prognostic factor for HCC [43]. The dominator in the process of reality engaging in HCC progression is SSRP1.

In HCC cells, SSRP1 controls both cell cycle and apoptosis [63]. When SSRP1 was overexpressed, cell migration and incursion increased. SSRP1 was inhibited, and cell migration and incursion decreased [64]. These findings suggested that SSRP1 played a role in reducing HCC cells' chemotherapeutic drug sensitivity. Though several theories have been suggested to explain it, the fundamental mechanism is still unknown. In the normal process of DNA replication, SSRP1 is an essential regulator. FACT interrelates with MCM helicase to conduct DNA unwinding on the nucleosome template. DNA replication is delayed when the FACT-MCM complex is interrupted [62, 65]. FACT has also been shown to influence the NF-B and p53 pathways in nearly all tumors, and its absence can lead to abnormal homologous recombination [66]. As a result, SSRP1 dysregulation triggers cancer genome instability, facilitating HCC progression in cells. SSRP1 has been identified as a key target in HCC for preventing metastasis and reversing opioid tolerance [65]. In a liver biopsy, SSRP1 can be assessed to predict the genetic activities of HCC. Multiple cancers have been identified to downregulate miR-497 and its tumor-suppressive activity, including head and neck, cervical, breast, lung, and prostate/ovarian cancer [67]. MYC activated DLG1-AS1 and the proliferation and migration of HCC through the SSRP1 axis (Figure 5). SSRP1 functions as an oncogene in HCC [68].

### 4.2. Colorectal Cancer and SSRP1

The lncRNA LOC101927746 inhibits colorectal cancer growth by overturning miR-584-3p and stimulating its target gene SSRP1 [69]. SSRP1 silencing inhibits colorectal cancer replication, migration, and incursion. It prevents the MAPK signaling pathway from being phosphorylated, which causes glioma cell production and metastasis. SSRP1 slows cancer cell growth and prevents erlotinib resistance by modulating the nuclear factor-kappa B signaling pathway. Disrupting the WNT signaling pathway, silencing SSRP1 with siRNA inhibits lung cancer progression, migration, and incursion. By inhibiting proliferation and encouraging apoptosis, SSRP1 silencing can activate the AKT signaling cascade. SSRP1 downregulation mediated by siRNA suppressed migration [28, 70]. In vivo, silencing SSRP1 inhibits the AKT signaling pathway, allowing downstream proteins to alter their expression. According to the researchers, SSRP1 inhibition prevents colorectal cancer proliferation and metastasis while also promoting apoptosis in vivo and vitro. The PI3K-AKT signaling pathway connects the survival and apoptosis of cells. In mammals, the serine/threonine kinase AKT (also known as protein kinase B), which has three isoforms (AKT1, 2, and 3), is a critical propagator of PI3K signaling [71, 72]. Metabolism, cell survival and its development, metastasis, and tumorigenesis are regulated by activated AKT, which phosphorylates a broad range of substrates. Silencing SSRP1 activated the AKT signaling pathway, which controls colorectal cancer [39]. SSRP1 silencing can trigger the AKT signaling pathway by preventing proliferation and encouraging apoptosis. Including siRNA, the migration was slowed by SSRP1 downregulation [73–75].

### 4.3. Ovarian Cancer and SSRP1

SSRP1 expression was more complex in ovarian cancer cells [73]. FACT provides a selective benefit to tumor cells under normal conditions and renders them more susceptible to curaxins cytotoxicity (Figure 6) [76]. Curaxins' tumor selectivity may be attributed to chromatin variations that allow tumor cells to have a higher demand for proof action than normal cells. FACT may have the same effect in normal tumor tissues. But NF-B-directed transcription can be more significant for tumor cells than normal cells. FACT's roles include histone dimer and tetramer attachment, including nucleosome remodeling in the vicinity of RNAPs.

The transcription of nucleosome-structured genes includes [48, 77] the presence of free soluble FACT. Owing to their near interaction with chromatin, curaxins promote FACT localization, resulting in the removal of soluble FACT. The affinity of truth for altered chromatin construction triggered by DNA intercalation of curaxins [78] is possible at the center of its “trapping” in chromatin. Curaxins-treated cells cause NF-B-dependent transcription to be suppressed by decreasing free FACT. It can also affect other transcriptional programs. The activation of p53 is also triggered by FACT binding to curaxins-impregnated chromatin. The SSRP1 HMG domain of FACT binds to twisted DNA [79]. This tends to prohibit CK2 from phosphorylating SSRP1's intrinsically disordered neighboring domain. CK2 does not have SSRP1 as a substrate and shifts its focus and phosphorylates p53 to Ser392. However, the existence of curaxins-induced changes in chromatin structure is uncertain. There was no significant curaxins-induced binding of FACT to nucleosomes in vitro assays [80]. Curaxins impregnation is insufficient because DNA crosslinks caused by cisplatin recruit FACT to twist DNA. In the context of chromatin, stronger/different DNA structure modifications are created [81, 82].

### 4.4. Gliomas and SSRP1

The MAPK signaling pathway is activated in over 88% of gliomas [83]. While the role of SSRP1 as a histone chaperone has been studied, little is known about its expression and possible molecular mechanism in glioma [59]. There was no discernible connection between SSRP1 expression and the patients' age or gender [54]. Based on cues, the MAPK pathway regulated many cellular programs, including differentiation, apoptosis, embryogenesis, and proliferation. The downregulation of SSRP1 led to a major reduction in phosphorylation of p38, ERK, and JNK, as well as overall p38 and ERK protein expression. The MAPK pathway could play a role in SSRP1's role in tumor progression [61]. The mesenchymal cells are at crossroads for SSRP1. It prevents adipocyte differentiation while fostering osteoblast differentiation. This phenomenon is greatly mediated by the modulation of the canonical Wnt/catenin signaling pathway having opposite effects on adipocyte and osteoblast differentiation being activated [53, 79]. siRNA inhibits U87 and U251 glioma cell proliferation by downregulation of SSRP1 [84]. p53 and NF-B are defined by their ability to change functions. Since it arbitrates the antitumor benefits of curaxins, FACT may be a future anticancer therapeutic goal. FACT expression is not apparent in Wi38 normal diploid fibroblasts and tumor cells [74, 75].

## 5. Concluding Remarks

SSRP1 is based on a chromatin transcription facilitated complex (also known as FACTp80) that replicates, transcribes, and repairs DNA. The cell differentiation stage is associated with SSRP1. In proliferation and undifferentiated cells, SSRP1 is highly articulated. SSRP1 is overexpressed in several tumor tissues but is underexpressed in mature tissues. In many cancer-related cases, elevated SSRP1 expression has been linked to metastasized tumors, making SSRP1 a potential prognostic marker and an anticancer target for tumor inhibition. Previous studies reported the emerging role of SSRP1 in various cancers, including HCC, colon, and ovarian cancer. However, there is still a long way ahead and tribulation in elucidating the complete role of SSRP1 in various human cancers. Furthermore, preclinical and clinical studies on the mechanism of SSRP1 will help explore the open new avenue for treating different human cancers.

## Figures and Tables

**Figure 1:** Major strategies in cancer therapy.

**Figure 2:** STRING network analysis showing SSRP1 (https://www.genecards.org/cgi-bin/carddisp.pl?gene=SSRP1).

**Figure 3:** Proposed scheme of regulating FACT complex subunits in mammalian cells. Reproduced with permission from [47].

**Figure 4:** DNA demethylation by DME requires SSRP1 function. Reproduced with permission from [58].

**Figure 5:** SSRP1 functions as an oncogene in HCC and activates the proliferation and migration of HCC. Reproduced with permission from [68].

**Figure 6:** (a) SSRP1 from the protein following curaxin treatment. (b) SSRP1 in cell lysates through Western blot analysis. (c) SPT16 and SSRP1 redistribution from the nucleoplasm to chromatin following curaxin treatment. (d) Anti-HMGB1 and anti-SSRP1 Western analysis. (e) Images of HT1080 cells infected with GFP-tagged SSRP1 and RFP-tagged histone H2B expression constructs. (f) Curaxin-induced depletion of soluble SSRP1 and SPT16 in vivo. (g) Western blot quantification of the data in (f). Reproduced with permission from [76].

## Data Availability

The data used to support the findings of this study are available from the corresponding author upon request.
